# Epigenetic Regulation of Methylation in Determining the Fate of Dental Mesenchymal Stem Cells

**DOI:** 10.1155/2022/5015856

**Published:** 2022-09-22

**Authors:** Hui Zhang, Hong Fu, Hongzhi Fang, Qing Deng, Hao Huang, Dingyu Hou, Miaomiao Wang, Quanzhou Yao, Qiqi Si, Rui Chen, Linke Li, Jie Weng, Tailin Guo, Mengyuan Wang

**Affiliations:** ^1^College of Medicine, Southwest Jiaotong University, Chengdu, Sichuan, China 610031; ^2^Department of stomatology, The Third People's Hospital of Chengdu, The Affiliated Hospital of Southwest Jiaotong University, Chengdu, Sichuan, China 610000; ^3^College of Materials Science and Engineering, Southwest Jiaotong University, Chengdu, Sichuan, China 610031; ^4^College of Analysis and Testing Center, Southwest Jiaotong University, Chengdu, Sichuan, China 610031; ^5^College of Life Science, Southwest Jiaotong University, Chengdu, Sichuan, China 610031; ^6^The Center of Obesity and Metabolic Diseases, Department of General Surgery, The Third People's Hospital of Chengdu & The Affiliated Hospital of Southwest Jiaotong University, No. 19 Yangshi Road, Chengdu, Sichuan, China 610031

## Abstract

Dental mesenchymal stem cells (DMSCs) are crucial in tooth development and periodontal health, and their multipotential differentiation and self-renewal ability play a critical role in tissue engineering and regenerative medicine. Methylation modifications could promote the appropriate biological behavior by postsynthetic modification of DNA or protein and make the organism adapt to developmental and environmental prompts by regulating gene expression without changing the DNA sequence. Methylation modifications involved in DMSC fate include DNA methylation, RNA methylation, and histone modifications, which have been proven to exert a significant effect on the regulation of the fate of DMSCs, such as proliferation, self-renewal, and differentiation potential. Understanding the regulation of methylation modifications on the behavior and the immunoinflammatory responses involved in DMSCs contributes to further study of the mechanism of methylation on tissue regeneration and inflammation. In this review, we briefly summarize the key functions of histone methylation, RNA methylation, and DNA methylation in the differentiation potential and self-renewal of DMSCs as well as the opportunities and challenges for their application in tissue regeneration and disease therapy.

## 1. Background

Dental mesenchymal stem cells (DMSCs) are multipotent progenitor cells with multilineage differentiation and self-renewal capability [1]. Recently, DMSCs have been obtained from periodontal, periapical, and pulpal tissue from permanent teeth [2]. DMSCs, a group of multipotent MSCs, contain dental follicle stem cells (DFSCs) [3], stem cells from alveolar bone (ABMSCs) [4], periodontal ligament stem cells (PDLSCs) [5], dental pulp stem cells (DPSCs) [6], stem cells from apical papillae (SCAPs) [7], stem cells from exfoliated deciduous teeth (SHED) [2], and stem cells from gingival tissue (GMSCs) (Figure 1) [8, 9]. DMSCs can differentiate into odontoblasts, chondrocytes, osteoblasts, adipocytes, neurons, and so on [10]. The excellent properties of DMSC make them play a critical role in tissue engineering and regenerative medicine [10–13].

Epigenetic regulation changes gene expression without altering the DNA sequence, meaning altering the gene expression potential stably during cell proliferation and differentiation [14]. Epigenetic mechanisms can promote appropriate biological behavior by postsynthetic modification of DNA or protein, making the organism adapt to developmental and environmental prompts by regulating gene expression [15, 16]. The main mechanisms of epigenetic regulation include methylation, ubiquitination, acetylation, and chromatin remodeling, which have been proven to exert a significant effect on the behavior of DMSCs, such as proliferation, self-renewal and differentiation potential [16]. Recently, there have been quantitative studies on the epigenetic underline of the biological and pathological processes in embryogenesis, development, and diseases. One important research topic is the effect of methyltransferase on DMSC fate, which includes DNA methylation, RNA methylation, and histone modifications [15, 17–19]. For example, both the histone demethylase lysine (K)-specific demethylase 6B (KDM6B) and lysine demethylase 2A (KDM2A) [20] participate in the osteogenic differentiation of DMSCs [21]. The histone demethylase KDM6B specifically demethylates dimethylation/trimethylation on lysine 27 of histone 3 (H3K27me2/3) and reactivates bone morphogenetic protein 2 (BMP2), which regulates osteogenic differentiation of DMSCs and plays a critical role in dental regeneration [22]. The silencing of KDM2A increases the H3K36me2 levels in the promoter of SFR2, which enhances the odontoblast differentiation potential of SCAPs [21]. 5-Aza-2′-deoxycytidine (5-Aza) is a DNA methyltransferase inhibitor that enhances the odontogenic differentiation of PDLSCs in DMSCs by decreasing the proliferation rate [4]. It was reported that DNA/histone methylation can regulate the osteogenic differentiation and proliferation of DPSCs [23].

In this review, we briefly summarize the key functions of histone methylation, RNA methylation, and DNA methylation in the differentiation potential and self-renewal of DMSCs as well as the opportunities and challenges for their application in tissue regeneration and disease therapy.

## 2. Characteristics and Clinical Potential of DMSCs

DMSCs have excellent properties, including self-renewal potency and multipotent differentiation capacity, which provide a new pathway for regenerative medicine [24]. Similar to stem cells (SCs), DMSCs are identified via cell surface markers, such as CD13, CD29, CD73, CD44, CD90, and CD105. Meanwhile, DMSCs negatively express hematopoietic markers, including CD14, CD19, CD34, CD45, CD11b, and HLR [25].

Among these DMSCs, DPSCs have attracted increasing attention in tissue regeneration due to their clonogenic efficiency and easy availability [26–29]. Moreover, DPSCs have the capacity for odontogenic and osteogenic differentiation to form dentin and bone tissues. PDLSCs exhibit multilineage differentiation potential and are isolated from human periodontal ligament. PDLSCs can be effectively applied in bone defect repair by modulating the immune microenvironment of the dental complex [30, 31]. A series of studies have demonstrated the multilineage differentiation potential and immunosuppressive property of DFSCs, and their unific characteristics make them applicable to the repair of periodontal defects and repression of inflammation in chronic inflammatory disease [32]. SCAPs can differentiate into osteoblasts, nerve cells, and adipocytes and exhibit immunosuppressive features [33]. SHED can regulate T cells and repress the function of T helper 17 cells to achieve immunomodulatory functions [34]. ABMSCs can regenerate new periodontium tissues and alveolar bone [35]. GMSCs can repair tongue muscle, mandibular, and calvaria defects as well as improve cementum, periodontal ligament, and alveolar bone regeneration [36, 37]. MSCs derived from the tooth germ (TGSCs) show excellent potential in osteogenic differentiation. In addition, TGSCs can differentiate into osteogenic, chondrogenic, neurogenic, and adipogenic cells [38]. TGSCs could be used in gingival tissue regeneration and therapy because of their easy accessibility and excellent differentiation potential [32, 39].

Currently, DMSCs can be applied to the therapy of oral diseases. DMSCs can reduce the inflammatory response by inhibiting the release of inflammatory cytokines to treat periodontal disease by promoting alveolar bone regeneration [1, 40]. Clinical studies found that DMSCs were able to regenerate compact substances of human mandibles, suggesting that DMSCs can be an attractive source of autologous transplantation for regenerative treatment [41, 42]. For example, PDLSCs with bone grafting material were transplanted into 16 defective teeth of three periodontitis patients, and all probing depths were reduced [43]. In bone tissue engineering, PDLSCs combined with tissue engineering scaffolds could regenerate alveolar bone in 30 periodontitis patients without significant adverse effects [44]. Autologous PDLSC niches were transplanted in 14 patients, and the probing pocket depth was reduced [45]. DPSCs combined with the scaffold material were implanted into the defect area of root furcation in two patients, and the results demonstrated that the periodontal defects were repaired [46]. The transplantation of DPSCs in five pulpitis patients promoted dentin formation safely and effectively [47]. Moreover, when DPSCs were mixed with support material and imputed into the bone defect of periodontitis patients, the bone defect was repaired, bone mineral density was increased, and the periodontal pocket depth was decreased in patients [48, 49].

## 3. Methylation Modifications of Epigenetics

Methylation modifications are the most common mechanism in complicated epigenetic processes and can regulate genes by changing the state of chromatin without altering the DNA sequence in cells [50], thus playing a vital role in gene expression, protein function, and RNA processing. Furthermore, methylation modifications include histone methylation, DNA methylation, and RNA methylation [51], which are dynamic processes regulated by methyltransferases and demethylases of histones, DNA, and RNA (Figure 2). These enzymes could control the fate of stem cells by mediating their pluripotency or differentiation [9, 52–56].

### 3.1. DNA Methylation

DNA methylation is a specific epigenetic mechanism that regulates gene expression and SC functions [57–60]. DNA methylation refers to the symmetrical addition of a methyl group on the 5-position of cytosine. This process is catalyzed by a group of enzymes, DNA methyltransferases (DNMTs), including DNMT1, DNMT3 L, DNMT3B, and DNMT3A [17, 61–66]. DNMTs at the cytosine residue at the 5-position in CpG dinucleotides transfer methyl groups of SAM (S-adenosylmethionine) to SAH (S-adenosylhomocysteine) and generate 5-methylcytosine (5-mC) [67]. DNA 5mC was discovered in 1948 and marked the prolusion of the consecutive research in epigenetic modification [66]. As one of the most common modification sites in eukaryotes [14, 68–70], it represses the binding of RNA polymerase and recruits binding proteins and thereby typically acts on epigenetic silencing of gene expression [18, 71]. DNA methylation status is stabilized via DNMTs and DNA demethylases. DNA demethylation is also vital during cellular proliferation and differentiation. 5-mC is converted to 5-hydroxy methylcytosine (5-hmC) via an oxidation reaction. This process is the first pathway of DNA demethylases and is mediated by the Ten–eleven translocation (TET) family, including TET1, TET2, and TET3 [61, 72]. Furthermore, thymine DNA glycosylase (TDG) could convert 5-hmC back to complete DNA demethylation and make the cytosine totally unmethylated, which is associated with the modification of G/T mismatches in DNA repair [17, 72] (Figure 3). Thus, DNA methylation plays a crucial role in the fate of SCs by gene regulation [59, 72].

### 3.2. Histone Methylation

DNA twines on histone proteins, including two dimers, H3/H4 and H2A/H2B, all of which compose a globular histone octamer and form the basic units of chromatin as nucleosomes [73]. The special structure of histones in eukaryotes exhibits a diversity of histone modifications, such as methylation, acetylation, phosphorylation, and ADP ribosylation [74]. Histone methylation induces alterations in chromatin structure by adjusting the density of nucleosomes, which regulates gene transcription [73] (Figure 4). Histone methylation mainly occurs at arginine and lysine residues of the tail in H3/4 and is mediated by protein lysine methyltransferases (PKMTs) and protein arginine methyltransferases (PRMTs) [74]. The lysine methylation sites, including histone H3 at lysine 4 (H3K4), H3K79, H3K36, H3K27, and H3K9, and trimethylation sites on lysine 4 of histone 3 (H3K4me3), lysine 27 of histone 3 (H3K27me3), and lysine 9 of histone 3 (H3K9me3) have been widely studied for the modification of genes [73, 75–77]. For instance, PRMTs catalyze arginine methylation. The yeast Dot1 and the mammalian homolog telomeric silencing 1 like (DOT1L) catalyze lysine methylation [78, 79]. Histone demethylases mainly contain the family of dioxygenase Jumonji-C (JmjC) domain proteins and the amine oxidases family of non-JmjC proteins, such as KDM6B and lysine-specific demethylase1 (LSD1) [20]. For example, KDM6B, a member of the oxidase family in the JmjC domain, can downregulate insulin-like growth factor binding protein 5 (IGFBP5) to enhance periodontal tissue regeneration by MSCs [80, 81]. LSD1 can reverse the methylation of H3K4, which may repress gene transcription [20, 76, 82]. Histone methylation has been widely studied and affects the fate of SCs [83, 84], such as cancer stem cells, adult tissue stem cells, and embryonic stem cells [19, 78, 83]. Additionally, histone methylation has the ability to regulate ESC differentiation and maintain the regeneration of neural stem cells and muscle stem cells [85]. They can also promote liver regeneration in animal experiments [86].

### 3.3. RNA Methylation

RNA methylation refers to the process of adding a methyl group to the methyl adenine of RNA [87]. RNA methylation includes N1-methyladenosine (m1A), N6-methyladenosine (m6A), 7-methyl guanosine (m7G), and 5-methylcytosineylation (m5C) modification of mRNA in eukaryotes [88–90]. As one of the most general RNA methylations, m6A RNA methylation refers to methylation of the adenosine (A) base at the nitrogen-6 site [87], and this has attracted more attention in recent years. RNA methylation is a reversible and posttranslational modification of RNA by catalysis of methyltransferase and demethylase [91]. m6A RNA methyltransferases catalyze RNA methylation and are known as “writers,” including methyltransferase-like protein 3 (METTL3), METTL14, and WTAP [92, 93]. The m6A RNA demethylase is known as an “eraser,” containing obesity-associated protein (FTO) and fat mass ALKB homolog 5 (ALKBH5), which regulates RNA demethylation [87, 89]. Readers include the YTH domain family (YTHDFs and YTHDCs) and IGF2BP1/2/3 family, which can directly bind to m6A to mediate downstream processes including mRNA export and mRNA translation [89–93] (Figure 5). m6A RNA methylation plays a critical role in biological processes by affecting gene translation, the DNA damage response, autophagy, stem cell proliferation, and fat formation [87, 89, 94–97]. For example, METTL3, as the most well-studied subunit of the m6A “writers,” could slow down the occurrence of chronic obstructive pulmonary disease and might promote tumor formation, migration, and invasion [98–100]. In addition, ALKBH5 has high expression in the embryonic stage and glioblastoma stem-like cells (GSCs), revealing that ALKBH5 may play an indispensable role in brain development and GSC proliferation [101–103]. FTO is associated with human diseases, including obesity, type 2 diabetes, coronary heart disease, and cancer [90, 104, 105].

## 4. Regulation of DMSCs by Methylation

Methylation has been proven to play a critical role in DMSCs, including PDLSCs, DFSCs, DPSCs, and SCAPs [4]. We briefly summarize some recent studies on methylation modifications and the clinical application potential of DMSCs.

### 4.1. PDLSCs

PDLSCs can be isolated from the periodontal ligament [106], and they can differentiate into alveolar bone, peripheral nerves, blood vessels, adipocytes, hepatocytes, and osteoblasts under specific conditions [21, 107]. PDLSCs have a positive effect on alveolar bone formation, which would rescue the loss of alveolar bone in periodontitis [108]. Furthermore, PDLSCs are used for repair of periodontal tissues and treatment of cartilage diseases in the regenerative medicine field [109, 110].

#### 4.1.1. Modification of PDLSCs by DNA Methylation

DNA methylation is a key regulatory component of epigenetic modification. Some papers have suggested that DNA methylation can regulate the fate of PDLSCs (Table 1). In the genomic analysis of DNA methylation, the DNA methylation of bone formation-related genes in PDLSCs was different from that in DPSCs and DFPCs. PDLSCs have lower methylation of osteogenic-related genes, such as runt-related transcription factor 2 (RUNX2), osteopontin (OPN), and alkaline phosphatase (ALP), leading to PDLSCs with better bone formation capacity in vivo [111]. Therefore, a better understanding of the DNA methylation of genes in PDLSCs is crucial to regulating osteogenic differentiation of PDLSCs and regeneration of periodontal tissue. For instance, the expression of RUNX2 was enhanced in the coculture of dedifferentiated fat cells (DFATs) with PDLSCs due to the downregulation of RUNX2 DNA methylation, which promoted the osteogenic potential of PDLSCs and DFATs [112]. Furthermore, hypermethylation of RUNX2 inhibits osteogenic differentiation of PDLSCs [113], and RG108 and 5-Aza, as DNMT1 inhibitors, could restore RUNX2 expression and increase the osteogenic potential of PDLSCs by eliminating the upregulated expression of DNMT1 in PDLSCs [114–116]. In addition, the destruction of the periodontium caused by lipopolysaccharide (LPS) leads to hypermethylation of RUNX2 in PDLSCs, which might directly hinder periodontal regeneration [115]. 5-Aza and RG108 may be potential therapies for periodontal diseases by restoring the hypermethylation of RUNX2.

In addition, a high-glucose (HG) environment inhibits the proliferation and differentiation of PDLSCs [117]. Increasing the expression of DNMT3A, DNMT3B, and DNMT1 in an HG environment causes DNA hypermethylation of osteogenic-related genes in PDLSCs, which has an inhibitory effect on the matrix mineralization of PDLSCs. However, 5-Aza reduces the DNA hypermethylation level and recovers the expression of osteogenic marker genes, such as ALP, OCN, OPN, and osterix (OSX, also called Sp7), thus rescuing matrix mineralization and stimulating osteogenic differentiation of PDLSCs [108]. In addition, tumor necrosis factor *α* (TNF-*α*) treatment of PDLSCs in an HG environment could cause PDLSCs to have lower cell viability [118]. The HG environment also inhibits the expression of DNMT1 protein while upregulating tumor necrosis factor-alpha receptor-1 (TNFR-1) due to the hypomethylation of CpG islands within the TNFR-1 gene in PDLSCs. However, SAM could downregulate TNFR-1 by increasing the methylation of TNFR-1 and then downregulating TNF-*α* and rescuing the cell viability of PDLSCs [118]. Modulation of DNA methylation by SAM or 5-Aza could regulate the viability and differentiation of PDLSCs in HG, which would be a potential treatment for periodontitis [108, 118].

On the other hand, inhibition of Ten–eleven translocation 1 (TET1) and Ten–eleven translocation 2 (TET2) could lead to the downregulation of the osteogenic and adipogenic capacity of PDLSCs, while the proliferation of PDLSCs could be enhanced [119]. In addition, Dickkopf-related protein-1 (DKK-1) exerts a negative effect on the Wnt pathway, thus inhibiting the immunomodulatory capacity of PDLSCs [120]. TET1 and TET2 binding to the DKK-1 promoter could maintain the hypomethylation of DKK-1 in PDLSCs and then inhibit the function of T cells induced by PDLSCs. Therefore, inhibition of TET1 and TET2 could result in hypermethylation of the DKK-1 promoter and significantly inhibit the expression of DKK-1 and in turn enhance the immunomodulatory capacity of PDLSCs [121]. Thus, downregulation of TET1 and TET2 may enhance the effect of PDLSC-mediated immunotherapy [119, 122].

#### 4.1.2. Modification of PDLSCs by Histone Methylation

Histone methylation is widely known to regulate the proliferation and differentiation of PDLSCs (Table 1). For example, downregulating the long noncoding RNA SNHG1 and upregulating Kruppel-like factor 2 (KLF2) both promote the osteoblastic differentiation of PDLSCs. SNHG1 inhibits the osteoblastic differentiation of PDLSCs by regulating H3K27me3 of KLF2 through zeste homolog 2 (EZH2) [123]. In addition, stress stimulation resulted in the upregulation of H3K27me3 signaling and the slight downregulation of transcription factor 2 (E2F), which induced transcriptomic changes and impaired the pluripotency of PDLSCs. Meanwhile, overexpression of EZH2 enhances the adipogenic differentiation of PDLSCs while suppressing osteogenic differentiation [110, 123]. Downregulation of EZH2 expression enhances ALP activity in PDLSCs induced by LPS [124]. Therefore, EZH2, as a histone methyltransferase, plays an important role in maintaining the differentiation of PDLSCs. Moreover, the in vitro and in vivo results showed that LPS induced the expression of H3K4me3 on inflammation-related genes. Inhibition of the protein lysine methyltransferase SET domain-containing 1B (SETD1B) led to the downregulation of H3K4me3, which decreased inflammatory genes and promoted osteogenic genes in PDLSCs [125]. In addition, upregulating the specific methyltransferase H3K36me3, known as SET domain-containing protein 2 (SETD2), can promote the osteogenic differentiation of PDLSCs [126]. Furthermore, histone methyltransferases such as EZH2, SETD1B, and SETD2 regulate the osteogenic differentiation of PDLSCs.

Histone methylation can be reversed by histone demethylases, such as lysine-specific demethylase 6A (KDM6A) and KDM6B. For instance, KDM6A promotes the expression of osteogenesis-related genes through the demethylation of H3K27me3 in the promoter region and facilitates the osteogenic differentiation of PDLSCs. Hence, overexpression of KDM6A enhances the osteogenic differentiation of PDLSCs [22, 127]. In addition, the absence of KDM6A elevates the level of H3K27me3 and decreases the expression of trimethylation on lysine 4 of histone 3 (H3K4me3), which ultimately suppresses the chondrogenic potential of PDLSCs [22]. However, treatment of PDLSCs with an inhibitor of EZH2 (EPZ-6438) rescued the impaired chondrogenesis of PDLSCs caused by the loss of KDM6A. Therefore, the regulation of KDM6A demethylation and the application of an EZH2 inhibitor potentially induces MSC-mediated cartilage regeneration in osteoarthritis [22]. Furthermore, Jiang and Jia found that miR-153-3 could inhibit the expression of KDM6A and the osteogenic differentiation of PDLSCs [127]. Therefore, downregulation of miR-153-3 or overexpression of KDM6A promotes the osteogenic differentiation of PDLSCs. These findings provide a new potential therapeutic application for PDLSCs in alveolar bone regeneration.

Moreover, both histone methyltransferases and demethylases regulate the fate of PDLSCs in an inflammatory environment. Knockdown of KDM6B inhibits the expression of RUNX2 and inflammatory factors in PDLSCs stimulated by LPS [124]. In addition, treatment of PDLSCs with LPS causes an increase in H3K27me3 on the promoters of OSX, RUNX2 and IL-1*β*. Therefore, LPS inhibits the proliferation and osteoblastic differentiation capacity of PDLSCs by increasing H3K27me3 on genes in PDLSCs. Glycoprotein nonmetastatic melanoma protein B (GPNMB) reduces LPS-induced apoptosis of PDLSCs as well as upregulates the expression of KDM6B, which could result in inhibiting the inflammatory response and apoptosis in periodontitis [128]. IGFBP5 can promote cell proliferation, chemotaxis, and migration in PDLSCs [80]. However, the deletion of the PR domain containing 9 (PRDM9) gene can upregulate IGFBP5 by increasing H3K4me3 of the IGFBP5 promoter, which enhances the transcription of IGFBP5 and promotes the proliferation, chemotaxis, and migration of PDLSCs [109]. Therefore, histone methylation has the ability to regulate the fate of PDLSCs via the regulation of different genes, such as RUNX2, GPNMB, and PRDM9.

### 4.2. DPSCs

DPSCs were first cultured in vitro by Gronthos et al. in 2000 [6]. DPSCs can differentiate into osteoblasts, cartilage heads, fats, blood vessels, odontoblasts, and so on [130]. Compared with other mesenchymal stem cells, DPSCs show better abilities, such as better odontoblast differentiation and viability. Nevertheless, DPSCs showed lower chondrogenic capacity [131–134]. Consequently, the differentiation ability and clinical application potential of DPSCs in regenerative medicine have attracted extensive attention [27].

#### 4.2.1. Modification of DPSCs by DNA Methylation

Numerous studies have also reported the function and regulation of DNA methylation in DPSCs (Table 2). DNMTs, such as DNMT1, DNMT3A, and DNMT3B, have an important effect on the differentiation of DPSCs [135]. DNA methylation mediated by these DNMTs can modulate odontogenic-related genes and calcium nodule formation. For instance, microRNA-675 (miR-675) regulates the odontogenic differentiation of DPSCs by suppressing DNMT3B-mediated methylation of distal-less homeobox 3 (DLX3) [136]. In addition, overexpression of lncRNA H19 (a classic long noncoding RNA) and miR-675 promotes the odontogenic differentiation potential of DPSCs by downregulating DNMT3B-mediated methylation of the DLX3 gene [137]. The methylation of KLF4 promoters mediated by DNMT1 is a transcription factor that can inhibit the odontoblast differentiation of DPSCs [138]. Kruppel-like factor 4 (KLF4) and SP1 enhance the odontoblastic differentiation of DPSCs as transcription factors [139, 140]. In contrast, RG108 and 5-Aza play a positive role in the differentiation of DPSCs. Inhibition of DNMT1 by RG108 increases KLF4, which improves the efficiency of odontoblast differentiation [138]. Hence, RG108, as a DNMT1 inhibitor, mediates the upregulation of SP1/KLF4 during the odontoblast differentiation of DPSCs. 5-Aza inhibits DNMT1 and BMP activity while promoting muscle-specific transcription factors in DPSCs. 5-Aza enhances the skeletal myogenic differentiation of DPSCs [141]. Furthermore, 5-Aza can promote myogenic differentiation and myogenic protein expression of DPSCs, and it can be used for the therapy of craniofacial muscles [142]. DPSCs with 5-Azax also increase ALP activity and calcified nodule formation, while odontogenic markers, including dentin matrix protein-1 (DMP-1), dentin sialo phosphoprotein (DSPP), RUNX2, DLX5, and OSX, are upregulated [143]. Therefore, 5-Azax has the ability to enhance the proliferation and differentiation of DPSCs by inhibiting DNA methylation. It was also found that pretreatment of DPSCs with 5-Aza after LPS stimulation reduced the m5C level of the TNF receptor-associated factor 6 (TRAF6) promoter [144]. As a result, inflammation-related signaling pathways were activated, such as the mitogen-activated protein kinase (MAPK) and nuclear factor-k-gene binding (NF-*κ*B) signaling pathways [144]. Therefore, DNA methylation plays a negative role in the regulation of DPSCs.

In contrast, DNA demethylase has a negative role in inflammatory responses of DPSCs induced by LPS. DPSCs stimulated by LPS increase the expression of TET2. TET2 knockdown downregulates the DNA hydroxymethylation of myeloid differentiation factor 88 (MyD88) promoter and inhibits the NF-*κ*B signaling pathway [145]. Therefore, understanding the regulation of DNA methylation is a potential treatment for pulpitis and periodontitis. Moreover, an in vitro experiment confirmed that the expression of TET1 was significantly increased during the proliferation of PDLSCs [146]. Therefore, the early differentiation and odontogenesis of DPSCs are associated with the level of TET1. Inhibiting the expression of TET1 in DPSCs decreases ALP activity and mineralized nodules during the odontogenic differentiation of DPSCs, which can ultimately inhibit the proliferation and differentiation of DPSCs [147]. During the odontogenic differentiation of DPSCs, deletion of TET1 leads to the downregulation of the family with similarity 20 member C (FAM20C) and enhances the mineralization of DPSCs [148]. FAM20C, also named dentin matrix protein 4 (DMP4), participates in the osteoblastic differentiation of DPSCs [149]. Therefore, TET1 enhances the odontoblastic differentiation of DPSCs by demethylating FAM20C.

#### 4.2.2. Modification of DPSCs by Histone Methylation

Three key markers of histone methylation, H3K4me3, trimethylation on lysine 9 of histone 3 (H3K9me3), and H3K27me3, play a significant role in the regulation of DPSCs [150] (Table 2). For instance, the promoters of early mineralization genes in DPSCs, such as RUNX2, DLX5, and MSX2, all contain H3K4me3 activity markers, which enhance the differentiation of DPSCs [150]. In addition, EZH2 catalyzes the methylation of H3K27me3, while KDM6B demethylates H3K27me3. The expression of EZH2 and H3K27me3 is decreased under inflammatory conditions [151], and the downregulation of EZH2 enhances the differentiation of DPSCs and suppresses the inflammatory response in DPSCs [152]. Moreover, EZH2 inhibition can enhance the osteogenic differentiation of DPSCs by activating *β*-catenin transcription and the Wnt signaling pathway [153]. Therefore, EZH2 inhibits osteogenic differentiation and promotes the inflammatory response. In contrast, KDM6B (also known as JMJD3), a member of the oxidase family of the JmjC domain, catalyzes the demethylation of H3K27me3 [154]. Under inflammatory conditions, the expression of KDM6B is increased, while H3K27me3 is decreased in DPSCs [151]. KDM6B activates odontogenic transcriptional genes and enhances the odontogenic differentiation of DPSCs by demethylating H3K27me3 of osteogenic genes, such as BMP2 and RUNX2 [154, 155]. Therefore, EZH2 and KDM6B could be applied to potential therapy in regenerating tooth structures. In addition, KDM5A is a histone demethylase (HDM), which is increased during the differentiation and early proliferation of DPSCs [156]. Knockdown of KDM5A enhances odontogenesis and mineralization in DPSCs by increasing H3K4me3 on the promoter of odontogenic marker genes [156]. Therefore, demethylation of H3K4me3 by KDM5A suppresses the dentin differentiation of DPSCs. These results indicated that the demethylation of KDM5A could be applied to dentin repair.

#### 4.2.3. Modification of DPSCs by RNA Methylation

There are also some reports about the regulation of m6A RNA methylation on osteogenic differentiation and proliferation of DPSCs (Table 2). m6A RNA methyltransferases (METTL3 and METTL14) and demethylases (FTO and ALKBH5) exist in PDLSCs [157]. The METTL3-mediated methylation of m6A RNA regulates the proliferation, migration, and differentiation of DPSCs [157, 158]. Bioinformatics analysis found that METTL3 was highly expressed in immature DPSCs and could regulate cell senescence and apoptosis [158]. Deletion of METTL3 resulted in activation of the p53 pathway in DPSCs and had a negative effect on the self-renewal of DPSCs. In addition, METTL3 mediates the expression of Polo-like kinase 1 (PLK1), a mitotic regulator that participates in cell cycle control and senescence apoptosis [158]. The results of in vivo experiments demonstrated that conditional knockout of METTL3 impaired the self-renewal, differentiation, and proliferation of DPSCs, thus damaging tooth root development [159]. The stimulation of LPS increases the expression of METTL3, while knockdown of METTL3 inhibits the expression of inflammation-related factors and inflammation-related signaling pathways, such as MAPK and NF-*κ*B signaling pathways [157]. Therefore, downregulating METTL3-catalyzed RNA methylation of m6A may inhibit the LPS-induced inflammatory response in DPSCs.

### 4.3. DFSCs

DFSCs can differentiate into alveolar bone, periodontal ligament, and root cementum. As the progenitor cells of some periodontal cell lineages [160–164], DFPCs can differentiate into chondrocytes, osteoblasts, adipocytes, and neural-like cells [4].

#### 4.3.1. Modification of DFSCs by DNA Methylation

DNMT1 can inhibit the osteoblastic differentiation of DFSCs by methylation of HOXA2 (Table 3). Overexpression of the lncRNA HOXA transcript antisense RNA myeloid 1 (HOTAIRM1) inhibits proliferation and enhances osteoblastic differentiation of DFSCs [78, 165, 166]. HOTAIRM1 restrains the DNMT1 and DNA methylation of HOXA2 catalyzed by DNMT1, which promotes the osteogenesis of DFSCs. HOTAIRM1 regulates the methylation state of the HOXA2 gene promoter by controlling DNMT1. Modulating the expression of the HOXA2 gene regulates the osteoblastic differentiation of DFSCs [78, 165, 166]. The upregulation of HOTAIRM1 may prevent the overmethylation of DFSCs from damaging periodontal tissue by inhibiting DNMT1.

#### 4.3.2. Modification of DFSCs by Histone Methylation

H3K4me3 is a marker that activates histone methylation, and H3K9me3 and H3K27me3 are markers of histone methylation that inhibit histone methylation. All of these markers can regulate the differentiation of DFSCs (Table 3). The promoters of the important factors that regulate osteogenic differentiation of DFSCs and early mineralization contain the active markers of H3K4me3. During osteogenic differentiation of DFSCs, H3K27me3 displays a prominent effect on DSPP and DMP-1, which are the promoters of dentin formation genes [111, 150, 167]. DFSCs can alter the expression of active H3K4me3, while PDLSCs and ABMSCs cannot. The H3K4me3 marker can turn to the H3K9me3 markers during osteogenic differentiation [167]. The expression of EZH2 and H3K27me3 can be decreased during the osteogenesis of DFSCs. EZH2 inhibits the osteogenesis of DFSCs by decreasing the H3K27me3 level of the Wnt gene promoter [168].

### 4.4. SCAPs

SCAPs were discovered in the apical papilla of human immature deciduous teeth, and they can differentiate into periapical tissue and pulp tissue [7, 169, 170]. SCAPs can exert vital effects on tooth development, especially in the odontoblasts in the root of the tooth [171]. Under suitable conditions in vitro, SCAPs can differentiate into adipocytes, hepatocytes, osteoblasts, neural cells, and odontoblasts [7, 169, 171].

#### 4.4.1. Modification of SCAPs by Histone Methylation

Recently, the histone methylation involved in the regulation of SCAP fate has attracted increasing attention (Table 4). KDM2A plays a negative role in osteogenic differentiation of SCAPs. The epiregulin (EREG) is a target of KDM2A (also known as FBXL11) that enhances osteogenic differentiation of SCAPs [172]. For instance, EREG is upregulated while KDM2A is downregulated during osteogenic differentiation of SCAPs. The KDM2A/BCL6 corepressor (BCOR) complex restrains histone H3 lysine 36/4 dimethylation (H3K36me2/H3K4me2) of the EREG promoter, which represses the transcription of the EREG promoter and inhibits osteogenic differentiation of SCAPs [172]. In addition, in SCAPs from oculofaciocardiodental (OFCD) syndrome patients, the methylation of H3K4 and H3K36 on the promotor of EREG is increased, which contributes to transcriptional activation of silent genes and enhancement of the osteogenic differentiation potential of SCAPs [173, 174]. However, overexpression of the histone demethylase KDM2A in SCAPs decreases EREG, which inhibits the expression of key transcription factors of bone-dentin differentiation, such as OSX and DLX2, and reduces the bone-dentin differentiation potential of SCAPs [172]. The upregulation of OSX and DLX2 promotes osteogenic differentiation of SCAPs by enhancing ALP activity and calcium mineralization [175]. In addition, secreted frizzled related protein 2 (SFRP2) inhibits NF-*κ*B signaling by repressing the Wnt/*β*-catenin signaling pathway in hypoxic and inflammatory conditions, and the expression of KDM2A in SCAPs is upregulated while the transcription of SFRP2 is inhibited and the methylation of H3K4me3 and H3K36me2 on the SCAP promoter is decreased [176]. Moreover, the study found that deletion of the demethylase KDM2A in SCAPs increased the methylation of H3K4 and H3K36 in the promoter of SFRP2 and inhibited their transcription. SFRP2 activated OSX and enhanced bone-dentin differentiation, while KDM2A exerted the opposite effect [177]. Therefore, KDM2A inhibits the osteoblastic differentiation of SCAPs by downregulating SFRP.

Lysine-specific demethylase 3B (KDM3B), lysine-specific demethylase 1A (KDM1A), mixed-lineage leukemia (MLL), and KDM6B also play critical roles in regulating the fate of SCAPs. KDM3B exerts a positive effect on osteoblastic differentiation of SCAPs by upregulating the expression of OCN, RUNX2, OSX, and DSPP. Moreover, KDM3B is involved in regulating the cell cycle to accelerate the proliferation of SCAPs [178]. In vitro, knockdown of KDM1A in SCAPs downregulates ALP activity and calcium mineralization of SCAPs. KDM1A combines with PLOD2 to form a protein complex that inhibits the bone-dentin differentiation of SCAPs [179]. MLL is a methylase of H3K4me3, KDM6B is the demethylase of H3K27me, and both promote odontogenic differentiation of SCAPs by upregulating Wnt5a [180–182]. The transcriptional activity of Wnt5a is regulated by H3K27me3 and H3K4me3. In addition, deficiency of the demethylase KDM6B enhances H3K27me3 and inhibits odontogenic differentiation [182].

## 5. Conclusion

Growing attention has been given to the differentiation, self-renewal, and regulation of DMSCs in the field of regenerative medicine [183–185]. For instance, DPSCs are used for the treatment of mandible defects and periodontal regeneration in chronic periodontitis patients [48, 186–188]. An ABMSC-based treatment strategy in the periodontal reconstruction of 27 patients enhanced periodontal tissue healing, periodontal bone reconstruction, reduction of probing pocket depth (mean ± SD, 0.75 ± 5.5 mm), and no adverse reactions after 12 months [189]. PDLSCs were filled into 10 patients with periodontal bone defects, and periodontal probing depth was reduced (3.2 ± 1.9 mm) while radiographic bone height was increased (2.3 ± 1.8 mm) in all 10 cases without serious adverse reactions in a clinical trial after 6 months [190]. The application of DMSCs is an opportunity for regenerative medicine, including the treatment of dental caries, pulp necrosis, periapical disease, and so on. However, the mechanism of the biology and regenerative ability of DMSCs requires further study.

Methylation modifications tightly and precisely regulate the fate of SC differentiation. For example, DNMT-mediated DNA methylation is essential for ESC differentiation [191]. Because of the lack of maintenance of DNMT1, extensive nonCpG methylation at CpA dinucleotides exists in ESCs [192]. Moreover, METTL3-/- mice showed abnormal differentiation of ESCs in vitro. METTL3 is a writer of m6A RNA methylation that can enhance the differentiation and reduce the self-renewal of ESCs [193, 194]. Furthermore, methylation modifications of SCs have been applied to clinical therapies. 5-AZA, as a DNMT inhibitor targeting brain cancer SCs, has been used in phase I trials to treat brain cancer [53]. It is also used to treat juvenile mononuclear leukemia (JMML) in conjunction with allogeneic hematopoietic stem cell transplantation (HSCT).

Recently, studies related to the cell proliferation and immune regulation of DMSCs by methylation modifications have attracted more attention [157, 158]. For example, the methyltransferase SETD1B catalyzed H3K4 histone trimethylation when DMSCs were stimulated by LPS, which increased H3K4me3 of gene promoters on IL-1*β* and IL-6, thus activating inflammatory signaling pathways and releasing inflammatory cytokines [125]. Knockdown of METTL3 and TET2 downregulated MyD88 and inhibited LPS-induced inflammatory responses in DPSCs [145, 157]. Therefore, understanding the regulation of methylation modifications on the immunoinflammatory responses involved in DMSCs in periodontitis contributes to further study of the mechanism of methylation on inflammation.

Increased DNA methylation and histone methylation have been reported to regulate the osteogenic differentiation of DMSCs, including PDLSCs, DPSCs, DFSCs, and SCAPs. More attention should be given to the regulation of RNA methylation in DMSCs. Additionally, further studies are also needed to study the methylation modification of DMSC proliferation, autophagy, apoptosis, and migration. Current studies still focus on animal experiments. For instance, DLX3 knockout in Wnt1-cre neural crest deletion mice causes major dentin defects [195]. METTL3 conditional knockout mice present molar root dysplasia [159]. Glucose inhibited the activation of DNMT1 and TNFR-1 [118], while TNF-*α* receptor p55-deficient mice showed less alveolar bone loss in periodontal tissues [196]. Kdm3C KO mice were more sensitive to LPS and showed increased alveolar bone loss [197]. Osr2-Cre; Ezh2fl/fl mice exhibited EZH2 participation in root patterning during molar root development [198]. In the future, more studies focusing on the methylation modifications of DMSCs, especially applications in tissue engineering and regulation of inflammation, are needed. These studies provide the basis for the therapy of oral disease and tissue regeneration applications.

## Figures and Tables

**Figure 1:** The different populations of dental tissue-derived stem cells and their distribution. Dental tissue-derived stem cells include dental mesenchymal stem cells and dental tissue-derived epithelial stem cells. DPSCs: dental pulp-derived stem cells; DFSCs: dental follicle stem cells; SCAPs: stem cells from apical papilla; PDLSCs: periodontal ligament stem cells; SHED: stem cells from exfoliated deciduous teeth GMSCs: stem cells from gingival tissue; ABMSCs: stem cells from the alveolar bone.

**Figure 2:** Methylation modifications' classification and main enzymes involved in methylation. Methylation modifications include DNA methylation, histone methylation, and RNA methylation. The enzymes include methyltransferase and demethylase.

**Figure 3:** Schematic representation of DNA methylation patterning. DNA methylation is exerted by DNA methyltransferases (DNMTs), including DNMT1, DNMT3L, DNMT3B, and DNMT3A. DNMTs at the cytosine residue at the 5-position in CpG dinucleotides transfer methyl groups and generate 5-methylcytosine (5-mC). DNA demethylation involves the successive oxidation of 5-mC to 5-hydroxymethylcytosine (5-hmC) by Ten–eleven translocation (TET) family, including TET1, TET2, and TET3. Thymine DNA glycosylase (TDG) could convert 5-hmC back to make the cytosine totally unmethylated.

**Figure 4:** Schematic representation of histone methylation and demethylation. DNA twines on histone proteins, including two dimers, H3/H4 and H2A/H2B, all of which compose a globular histone octamer and form the basic units of chromatin as nucleosomes. Histone methylation mainly occurs at arginine and lysine residues of the tail in H3/4 and is mediated by methyltransferases and histone demethylation is regulated by demethylases. Histone methylation can affect the spatial structure of chromatin by affecting the structure of nucleosomes and thus regulating the expression activity of genes. The nucleosome structure usually becomes crowded by adding methyl group (Me) from arginine and lysine residues of the tail, which making it difficult for gene segments to be transcribed, so gene expression is silenced. In contrast, the demethylation of histone usually could induce the open histone structure by removing methyl group (Me) from arginine and lysine residues of the tail, which expose the transcription factor binding sites and regulates the transcriptional activation of genes.

**Figure 5:** The dynamic and reversible processes of m6A methylation. m6A RNA methylation is mainly regulated by its “writers,” “erasers,” and “readers.” Writers refer to the m6A methylase complex including METTL3, METTL14, and WTAP. Erasers are m6A demethylases involving FTO and ALKBH5. Readers include the YTH domain family (YTHDFs and YTHDCs) and IGF2BP1/2/3 family. “Writers” deposit m6A methylation on RNAs, while “erasers” remove the m6A marks. “Readers” can directly bind to m6A to mediate downstream processes including mRNA export and mRNA translation.

**Table 1:** Methylation and demethylation in PDLSCs.

Methylated modification	Epigenetic modifiers	Epigenetic marks	Functions
DNA methylation	RG108	DNMT inhibitor	The hypomethylation of RUNX2 promoted osteogenic potential [116].
	5-Aza	DNMT inhibitor	Down-regulating expression of DNMT1, stimulating osteogenic differentiation [108, 113, 115, 117, 118].
	SAM	Methyl-donor	Rescuing the cell viability and increasing the methylation of TNFR-1 [118].
DNA demethylation	TET1/2	DNA demethylases	Enhancing differentiation while inhibiting immune regulation [119–122, 129].
Histone methylation	EZH2	H3K27me3	Inhibiting the osteogenic differentiation [110, 123, 124, 129].
	SETD1B	H3K4me3	Downregulating the release of inflammatory factors from PDLSCs stimulated by LPS [125].
	SETD2	H3k36me3	Promoting the osteogenic differentiation [126].
Histone demethylation	KDM6A	H3K27me3, H3K4me3	Enhancing the osteogenic differentiation [22, 127].
	EPZ-6438	EZH2 inhibitor	Rescuing the chondrogenic potential of PDLSCs by decreased H3K27me3 [22].
	KDM6B	H3K27	Enhancing periodontitis inflammatory response and apoptosis [124, 128].
		H3K4me3	Promoting potential of proliferation, chemotaxis and migration [109].

**Table 2:** Methylation and demethylation in DPSCs.

Methylated modification	Epigenetic modifiers	Epigenetic mark	Function
DNA methylation	DNMT3A	DNMTs	Regulating the odontogenic differentiation [135].
	DNMT3B	DNMTs	Enhancing the odontogenic differentiation of DPSCs by inhibiting DNMT3B-mediated-methylation of DLX3 [135–137].
	DNMT1	DNMTs	The methylation of KLF4 promoters by DNMT1 inhibited the odontoblast differentiation of DPSCs [138].
	RG108	DNMT inhibitor	Improving the efficiency of odontoblast differentiation [138].
	5-Aza	DNMT inhibitor	Inhibiting inflammation while enhancing myogenic differentiation and odontogenic differentiation [141–144].
DNA demethylation	TET2	DNA demethylases	TET2 knockdown downregulates MyD88 promoter methylation and inhibits LPS-induced inflammatory responses in DPSCs [145].
	TET1	DNA demethylases	Enhancing self-differentiation and odontogenesis [146–148].
Histone methylation		H3K4me3	Enhancing the differentiation [150].
	EZH2	H3K27me3	Reducing H3K27me3 expression increased that of KDM6B in DPSCs under inflammation and inhibition of EZH2 can activate *β*-catenin transcription and Wnt signaling pathway to promote the osteogenic differentiation [151–153].
Histone demethylation	KDM6B	H3K27me3	Removing H3K27me3 methylation, activating odontogenic transcriptional gene activation and enhancing the odontogenic differentiation [151, 154, 155].
	KDM5A	H3K4me3	Demethylation of H3K4me3 suppresses the dentin differentiation of DPSCs [156].
RNA methylation	METTL3	m6A	Regulating the proliferation, migration, differentiation, root formation, cell senescence, and apoptosis. Knockdown of METTL3 reduces the expression of inflammation-related factors and activation of signaling pathways induced by LPS [158/157, 159/158, 160/159].
RNA demethylation	METTL14	m6A	Expressing in PDLSCs [158/157].
	FTO	m6A	Expressing in PDLSCs [158/157].

**Table 3:** Methylation and demethylation in DFSCs.

Methylated modification	Epigenetic modifiers	Epigenetic marks	Functions
DNA methylation	DNMT1	DNA methyltransferases	Inhibiting osteogenesis [78, 166].
	5-Aza	DNMT inhibitor	Promoting osteogenesis [78, 166].
Histone methylation		H3K4me3, H3K9me3	H3K4me3 marker will switch to the H3K9me3 marker during osteogenic differentiation [167].
	EZH2	H3K27me3	EZH2 inhibits the osteogenesis of DFSCs by reducing H3K27me3 expression of Wnt gene promoter [111, 150, 168].

**Table 4:** Methylation and demethylation in SCAPs.

Methylated modification	Epigenetic modifiers	Epigenetic marks	Functions
Histone demethylation	KDM2A	H3K36me2, H3K4me2	Inhibiting osteogenic differentiation [172–177].
	KDM3B	H3K9me2	Exerting a positive impact on osteogenic differentiation of SCAPs and regulating the cell cycle to accelerate the proliferation of SCAPs [178].
	KDM1A	H3K4me2/1, H3K9me2/1	KDM1A forms a protein complex with PLOD2 to inhibit the bone-dentin differentiation [179].
	MLL	H3K4me3	Promoting odontogenic differentiation of SCAPs by upregulating Wnt5a [182].
	KDM6B	H3K27me3	Loss of the demethylase KDM6B increases H3K27me while inhibits odontogenic differentiation [182].

## Abbreviations

DMSCs: Dental mesenchymal stem cells
DPSCs: Dental pulp stem cells
DFSCs: Dental follicle stem cells
PDLSCs: Periodontal ligament stem cells
SCAPs: Stem cells from apical papillae
SHED: Stem cells from exfoliated deciduous teeth
ABMSCs: Stem cells from alveolar bone
GMSCs: Stem cells from gingival tissue
KDM6B: Lysine (K)-specific demethylase 6B
KDM2A: Lysine demethylase 2A
H3K27me2/3: Demethylation/trimethylation on lysine 27 of histone 3
BMP2: Bone morphogenetic protein 2
5-Aza: 5-Aza-2′-deoxycytidine
SCs: Stem cells
TGSCs: MSCs derived from the tooth germ.
SAM: S-Adenosyl methionine
SAH: S-Adenosyl homocysteine
DNMTs: DNA methyltransferases
HSCs: Hematopoietic stem cells
TET: Ten–eleven translocation
TET1: Ten–eleven translocation 1
ESCs: Embryonic stem cells
TET2: Ten–eleven translocation 2
5-mC: 5-Methylcytosine
5-hmC: 5-Hydroxy methylcytosine
TDG: Thymine DNA glycosylase
PRMTs: Protein arginine methyltransferases
PKMTs: Protein lysine methyltransferases
DOT1L: Telomeric silencing 1 like
JmjC: Jumonji C-terminal
LSD1: Lysine-specific demethylase 1
IGFBP5: Insulin-like growth factor binding protein 5
H3K4: Histone H3 at lysine 4
m1A: N1-Methyladenosine
m6A: N6-Adenine methylation
m7G: 7-Methyl guanosine
METTL3/14: Methyltransferase-like protein 3/14
FTO: Obesity-associated protein
ALKBH5: Fat mass alkB homolog 5
GSCs: Glioblastoma stem-like cells
RUNX2: Runt-related transcription factor 2
ALP: Alkaline phosphatase
OPN: Osteopontin
DFATs: Dedifferentiated fat cells
LPS: Lipopolysaccharide
HG: High glucose
EZH2: Enhancer of zeste homolog 2
OSX: Osterix
E2F: Transcription factor 2
TNF-*α*: Tumor necrosis factor *α*
SETD1B: SET domain-containing 1B
TNFR-1: Tumor necrosis factor-alpha receptor-1
DKK-1: Dickkopf-related protein-1
hnRNPL: Heterogeneous nuclear ribonucleoprotein L
KLF2: Kruppel-like factor 2
SETD2: SET domain-containing protein 2
KDM6A: Lysine- specific demethylase6A
H3K4me3: Trimethylation on lysine 4 of histone 3
GPNMB: Glycoprotein nonmetastatic melanoma protein B
PRDM9: PR domain containing 9
miR-675: MicroRNA-675
DLX3: Distal-less homeobox 3
KLF4: Kruppel-like factor 4
DSPP: Dentin sialophosphoprotein
DMP-1: Dentin matrix protein-1
NF-*κ*B: Nuclear factor-*κ*B
TRAF6: TNF receptor-associated factor 6
MAPK: Mitogen-activated protein kinase
MyD88: Myeloid differentiation factor 88
FAM20C: Family with sequence similarity 20, member
H3K9me3: Trimethylation on lysine 9 of histone 3
DMP4: Dentin matrix protein 4
HDMs: Histone demethylases
EREG: Epithelial regulatory factor
HOTAIRM1: lncRNA HOXA transcript antisense RNA myeloid 1
PLK1: Polo-like kinase 1
H3K36me2/H3K4me2: Histone H3 lysine 36/4 dimethylation
BCOR: BCL6 corepressor
OFCD: Oculofaciocardiodental
SFRP2: Secret frizzled-related protein 2
KDM3B: Lysine-specific demethylase 3B
KDM1A: Lysine-specific demethylase 1A
MLL: Mixed-lineage leukemia
JMML: Juvenile mononuclear leukemia
HSCT: Hematopoietic stem cell transplantation.
